The article "A novel bacterial isolate Stenotrophomonas maltophilia as living factory for synthesis of gold nanoparticles" was retracted in 2009. Reason: duplicate publication.

# A novel bacterial isolate *Stenotrophomonas maltophilia *as living factory for synthesis of gold nanoparticles

**DOI:** 10.1186/1475-2859-8-39

**Published:** 2009-07-20

**Authors:** Yogesh Nangia, Nishima Wangoo, Nisha Goyal, G Shekhawat, C Raman Suri

**Affiliations:** 1 Institute of Microbial Technology (CSIR), Sector 39-A, Chandigarh 160036, India; 2 Institute of Nanotechnology, Northwestern University, Evanston, IL, USA

## Abstract

**Background:**

The synthesis of gold nanoparticles (GNPs) has received considerable attention with their potential applications in various life sciences related applications. Recently, there has been tremendous excitement in the study of nanoparticles synthesis by using some natural biological system, which has led to the development of various biomimetic approaches for the growth of advanced nanomaterials. In the present study, we have demonstrated the synthesis of gold nanoparticles by a novel bacterial strain isolated from a site near the famous gold mines in India. A promising mechanism for the biosynthesis of GNPs by this strain and their stabilization via charge capping was investigated.

**Results:**

A bacterial isolate capable of gold nanoparticle synthesis was isolated and identified as a novel strain of *Stenotrophomonas malophilia *(AuRed02) based on its morphology and an analysis of its 16S rDNA gene sequence. After 8 hrs of incubation, monodisperse preparation of gold nanoparticles was obtained. Gold nanoparticles were characterized and found to be of ~40 nm size. Electrophoresis, Zeta potential and FTIR measurements confirmed that the particles are capped with negatively charged phosphate groups from NADP rendering them stable in aqueous medium.

**Conclusion:**

The process of synthesis of well-dispersed nanoparticles using a novel microorganism isolated from the gold enriched soil sample has been reported in this study, leading to the development of an easy bioprocess for synthesis of GNPs. This is the first study in which an extensive characterization of the indigenous bacterium isolated from the actual gold enriched soil was conducted. Promising mechanism for the biosynthesis of GNPs by the strain and their stabilization via charge capping is suggested, which involves an NADPH-dependent reductase enzyme that reduces Au^3+ ^to Au^0 ^through electron shuttle enzymatic metal reduction process.

## Background

Synthesis of GNPs and subsequent linkage to biomolecules has contributed immensely in various life sciences related applications such as drug-delivery, gene transfer, bioprobes in cell and tissue analysis for visualization of micro- and nano-objects, and for observation of the biological processes at nano-scale etc. [1-5]. These nanoparticles, in general, are synthesized using a number of synthetic procedures in various polar and non-polar media [6-8]. Recently, there has been tremendous excitement in the study of nanoparticles synthesis by using some natural biological system. This has led to the development of various biomimetic approaches for the growth of advanced nanomaterials. Microorganisms, such as bacteria, yeast and fungi, are known to produce inorganic materials either intra- or extracellularly [9-12]. These microorganisms play an important role in remediation of metals through reduction of metal ions. Some of these microorganisms can survive and grow even at high metal ion concentrations. They are often exposed to extreme environmental conditions, forcing them to resort to specific defense mechanisms to quell such stresses, including the toxicity of foreign metal ions or metals [13]. The toxicity of metal ions is reduced or eliminated by changing the redox state of the metal ions and/or precipitation of the metals intracellularly, thus, forming the basis of the synthesis of nanoparticles [14]. However, the actual mechanism for the biosynthesis of GNPs by different microorganisms and their stabilization via charge capping is still not well understood. It was shown in one of the earlier studies that the possible mechanism of biosynthesis of silver nanoparticles might involve the reduction of silver ions due to the electron shuttle enzymatic metal reduction process. The enzyme involved in the synthesis of silver nanoparticles may be nitrate reductase present in microorganism, which may be induced by the nitrate ions and reduced silver ions to metallic silver [15]. Duran *et al *also suggested the possible mechanism of biosynthesis of silver nanoparticles by *Fusarium oxysporum *strains (fungi). They proposed the involvement of enzymatic electron shuttle relationship for the formation of Ag^+ ^ions and the subsequent formation of silver nanoparticle [16]. Although there are reports on the biochemical steps involved in metallic nanoparticles synthesis by microorganisms [17-20], there are virtually no reports available which may elucidate enzymatic basis of gold nanoparticle synthesis by *Stenotrophomonas maltophilia*.

In this paper, we report the rapid synthesis of GNPs by *Stenotrophomonas maltophilia *(Acc No GQ220749), a novel bacterial strain isolated from soil samples from the Singhbhum gold mines (located in the Jharkhand state of India). A possible mechanism of biosynthesis of gold nanoparticles from gold chloride (HAuCl_4_) involves the role of specific NADPH-dependent reductase enzyme present in the organism that converts Au^3+ ^to Au^0 ^through electron shuttle enzymatic metal reduction.

## Results and discussion

### Isolation and characterization of strain capable of synthesisizing gold nanoparticles

Pure colonies isolated from the gold enriched soil were characterized for their morphological and physiological characteristics by various biochemical tests using the Bergeys Manual of Determinative Bacteriology [21] as summarized in Table 1. The screened strain is aerobic, motile, mucoid and yellow in Nutrient Agar medium (Himedia Labs, India). SEM micrographs revealed that the cells of strain AuRed02 are oval shaped, with discrete lipopolysaccharides layers on its surface causing the bacteria to glue to each other as evident from SEM imaging (Fig. 1). No production of acid was noted from the selected carbohydrates such as adonitol, arabinose, fructose, galactose, inositol, inulin, lactose, mannitol, mannose, rhamnose, sorbitol and xylose. The isolated strain named as AuRed02 produced acid from maltose, dextrose and trehalose, showing typical characteristics of *Stenotrophomonas maltophilia*. The strain gave a positive lipolytic activity and was able to utilize citrate as a carbon source.

**Table 1:** Biochemical tests of the isolated strain *Stenotrophomonas maltophila *AuRed02

Gram staining	Negative
Catalase test	Positive

Citrate test	Positive

Oxidase test	Negative

Glucose o/f test	Negative

Methyl red test	Negative

Gelatin test	Positive

**Carbohydrate utilization tests**	

Adonitol	Negative

Arabinose	Negative

Cellobiose	Positive

Dextrose	Positive

Fructose	Negative

Galactose	Negative

Inositol	Negative

Inulin	Negative

Lactose	Negative

Maltose	Positive

Mannitol	Negative

Mannose	Negative

Rhamnose	Negative

Salicin	Positive

Sorbitol	Negative

Sucrose	Positive

Trehalose	Positive

Xylose	Negative

**Figure 1:** **SEM image of *Stenotrophomonas maltophilia *cells**. Scale bar corresponds to 1 μm. The cells were imaged after reaction with gold chloride solution for 8 hrs.

The 16S rDNA sequence analysis revealed that strain AuRed02 clustered homologue being *Pseudomonas Sp. *(Acc. No. FJ211222). At species level, strain AuRed02 shows the highest level of sequence similarity with *Stenotrophomonas maltophilia *strain: BL-15 (99%) (AB194325) as shown in phylogenetic tree (Fig. 2).

**Figure 2:** **Phylogenetic tree made in MEGA 3.1 software using Neighbor joining method**.

### Characterization of gold nanoparticles synthesized by *Stenotrophomonas maltophilia*

A solution of gold chloride in a suspension of cell mass of *Stenotrophomonas maltophilia *changed progressively from light yellow to cherry red at temperature 25°C showing formation of gold nanoparticles. Control experiments, without the addition of biomass as well as with heat-killed cells, showed no change in color of suspension (Fig. 3a) confirming the formation of GNPs in the presence of biomass only. The kinetics of the reaction was studied using UV-vis spectroscopy by recording spectra from the colloidal gold solutions obtained after disrupting the cells, which were resuspended with HAuCl_4 _solution for different time intervals. The spectra revealed a strong absorption at nearly 530 nm after 8 hrs of incubation at 25°C, gradually showing a red shift with time at 25°C (Fig 4 curves bottom to top). The intense plasmon resonance band indicated the formation of spherical gold nanoparticles of approximately 40 nm in diameter [18]. Size distribution of GNPs was confirmed by coating a drop of the supernatant solution of disrupted cell suspension by TEM imaging. The images demonstrate gold nanoparticles possessing an average diameter of 40 nm (± 15%) as depicted in (Fig. 3b). Cryo TEM imaging of the thin sections of stained AuRed02 strain after reacting the biomass with gold chloride solution for 8 h showed the presence of gold nanoparticles on the inner cytoplasmic membrane (see Additional file 1, S1). It is likely that some gold ions (Au^3+^) cross the cell barrier through ion-transport channel and are reduced by the enzymes present on the cytoplasmic membrane and within the cytoplasm. Energy dispersive spectroscopy analysis (EDS) confirmed the presence of gold nanoparticles in the suspension. The spectra (Fig. 3c) present major Au peaks at approximately 2 keV besides several other peaks of C, O, and Si which might be due to the chemical composition of the sample substrate used in the EDS analysis. These results show that the strain *Stenotrophomonas maltophilia *could effectively synthesize GNPs of different sizes by resuspending the biomass for different time intervals in the presence of HAuCl_4 _(Fig. 4). The colored solution of GNPs remained stable for more than 2-weeks of storage at 4°C indicating the capping of GNPs with some charged groups. FTIR analysis of these GNPs further confirmed the capping of GNPs by phosphate groups (900 cm^-1^) (see Additional file 1, S2).

**Figure 3:** **(A) GNPs synthesised by *Stenotrophomonas maltophilia *(tube A)**. Control experiments: gold chloride incubated without the biomass (tube B) and with heat-killed cell mass (tube C). (B) TEM image recorded from a drop-coated film of disrupted cell suspension. Scale bar corresponds to 200 nm. (C) Energy Dispersive Spectra of synthesized GNPs showing Au peaks as major constituent.

**Figure 4:** **UV-vis spectra of GNPs solutions prepared by resuspending the biomass of Stenotrophomonas maltophilia for different time intervals in the presence of 1 mM HAuCl_4_**.

### Promising mechanism aspects of biosynthesis by *Stenotrophomonas maltophilia*

In microorganisms, the possible mechanisms of resistance against metal ions usually involve biosorption, bioaccumulation, extra-cellular complexation, efflux system, alteration of solubility and toxicity via reduction or oxidation [22]. Our study suggested that the biosynthesis of GNPs and their stabilization via charge capping in *Stenotrophomonas maltophilia *involved NADPH-dependent reductase enzyme that converts Au^3+ ^to Au^0 ^through electron shuttle enzymatic metal reduction process. For further confirmation, biomass was incubated with varying concentrations of NADPH (from 0.05 mM to 0.8 mM NADPH) and change in color of solution was monitored spectrophotometrically (Fig 5a) and visually (Fig. 5b). Control experiments, without the addition of either cell free extract (C1) or cell free extract without NADPH (C2), showed no change in color of suspension. However, addition of NADPH in the cell free extract at varying concentrations (C3 to C7) showed the synthesis of GNPs with gradual increase in color intensity (Fig. 5b). This confirms the formation of GNPs only in the presence of both biomass and NADPH. Zeta potential measurements of the GNPs showed a peak at -16.7 mV (see Additional file 1, S3), suggesting capping of GNPs by negatively charged phosphate ions from NADP. Based on these experimental findings, a schematic representation of the potential mechanism of gold nanoparticles synthesis by *Stenotrophomonas maltophilia *through enzymatic reduction is proposed (Fig. 6). The enzyme involved in the synthesis of metal nanoparticles may be a specific reductase present in microorganism, which may be induced by the specific ions and reduced metal ions to metallic nanoparticles.

**Figure 5:** **(A) UV-vis spectra of GNPs synthesis by adding different concentrations of NADPH in the solution of suspended biomass along with HAuCl_4 _(C3 to C7) and (B) shows the GNPs synthesis by adding different concentrations of NADPH in the solution of suspended biomass along with HAuCl_4 _(tubes C3 to C7)**. In controls (C1 and C2), either cell mass (C1) or NADPH (C2) was not added.

**Figure 6:** **Proposed synthesis mechanism of GNPs by *Stenotrophomonas maltophilia *through enzymatic reduction**.

## Conclusion

The process of synthesis of well-dispersed nanoparticles using a highly efficient microorganism *Stenotrophomonas maltophilia *has been reported in this study leading to the development of an easy bioprocess for synthesis of GNPs of desired size and shape. The results presented demonstrate that a specific NADPH-dependent enzyme present in the isolated strain reduces Au^3+ ^to Au^0 ^through an electron shuttling mechanism leading to the synthesis of nearly monodispersed GNPs. This green route of biosynthesis of GNPs is a simple, economically viable and an eco-friendly process.

## Methods

### Isolation and characterization of bacteria from the gold enriched soil

Soil samples from the gold enriched sites near famous Singhbhum gold mines, Jharkhand state, India were used as inoculum, serially diluted and plated onto Nutrient Agar media (Himedia, India). The plates were incubated at 30°C for 24 hrs. The colonies obtained were further subcultured on Nutrient Agar supplemented with 1 mM HAuCl_4 _(Sigma, India) and incubated at 30°C for 24 hrs. In one of the isolates, the light yellow color of HAuCl_4 _changed to wine red indicating that the organism was utilizing HAuCl_4 _for the synthesis of GNPs. The morphological and physiological characterization of the selected isolate was carried out by biochemical tests using the Bergeys Manual of Determinative Bacteriology [21]. The cell morphology was investigated using Zeiuss-EVO 40 scanning electron microscope (SEM). Further characterization of isolate was done by means of 16S rRNA gene analyses [23]. The 16S rDNA sequencing was done by M/s Bangalore Genei, India.

To obtain stable gold nanoparticles, the conditions of the characterized isolate were optimized for different concentrations of gold chloride, production media, temperature, pH and time. The characterized isolate was inoculated into 50 ml sterile Nutrient Broth (NB) and subsequently 1 gm of wet biomass was harvested after 16 hrs of incubation. The biomass obtained was washed thrice with deionised water (pH 7.0) and added to a 100 ml Erlenmeyer flask containing 1 mM gold chloride solution prepared in de-ionized water spiked with 400 mg Yeast Extract. The Erlenmeyer flasks were incubated at 25°C for 8 hrs to isolate the nearly monodisperse spherical gold nanoparticles. To isolate the pure GNPs, cells were disrupted using 0.2% (v/v) Triton X-100. The disrupted samples were centrifuged at 3500 rpm for 15 min at 4°C and washed thrice with deionized water to remove cell-debris. The supernatant was used for the characterization of GNPs.

### Biosynthesis of gold nanoparticles and their characterization

To determine the peak time-point of maximum gold nanoparticles synthesis, the absorption spectra of the supernatants were taken at different time intervals and recorded using a Hitachi U2800 spectrophotometer. TEM studies were carried out using Jeol 2100 microscope operating at 120 kV accelerating voltage. Samples were prepared by placing a drop of GNPs solutions on carbon-coated TEM grids. The films on the TEM grids were allowed to dry for 5 min at room temperature before analysis. Energy dispersive spectroscopy analysis (EDS) was carried out to confirm the synthesis of gold nanoparticles using FEI E-SEM Quanta 200. Particle size and charge distribution (zeta potential) was analyzed using dynamic light scattering system (Beckman Coulter, USA) by illuminating the colloidal gold solution with He-Ne Laser (633 nm) in a sample cell.

## Competing interests

The authors declare that they have no competing interests.

## Authors' contributions

YN and NG carried out the isolation and characterization work of bacterial isolate described in the paper. NW took part in the characterization of gold nanoparticles and described the mechanism aspects of biosynthesis. GS did all TEM analysis and CRS coordinated the research as well as the manuscript preparation. All authors read and approved the final manuscript.

## Supplementary Material

Additional file 1 S1: Cryo TEM imaging of the thin sections of stained AuRed02 strain; S2: FTIR analysis of GNPs; S3: Zeta potential measurements of the GNPs. Click here for file
